This article has been retracted.

# Novel lncRNA AL033381.2 Promotes Hepatocellular Carcinoma Progression by Upregulating PRKRA Expression

**DOI:** 10.1155/2022/1125932

**Published:** 2022-01-07

**Authors:** Feiran Wang, Lirong Zhu, Qiang Xue, Chong Tang, Weidong Tang, Nannan Zhang, Chen Dai, Zhong Chen

**Affiliations:** ^1^Medical College of Nantong University, Nantong, Jiangsu 226000, China; ^2^Department of General Surgery, Affiliated Hospital of Nantong University, Nantong, Jiangsu 226000, China; ^3^Department of Radiotherapy, Affiliated Hospital of Nantong University, Nantong, Jiangsu 226000, China; ^4^Department of General Surgery, Affiliated Hospital 2 of Nantong University, Nantong, Jiangsu 226000, China; ^5^Institute of Organ Transplantation, Tongji Hospital, Tongji Medical College, Huazhong University of Science and Technology; Key Laboratory of Organ Transplantation, Ministry of Education, NHC Key Laboratory of Organ Transplantation, Key Laboratory of Organ Transplantation, Chinese Academy of Medical Sciences, Wuhan, Hubei 430030, China

## Abstract

Hepatocellular carcinoma (HCC) is a common malignant tumor that is characterized by aggressiveness and poor prognosis. Accumulating evidence indicates that oxidative stress plays a crucial role in carcinogenesis, whereas the potential mechanism between oxidative stress and carcinogenic effects remains elusive. In recent years, long noncoding RNAs (lncRNAs) in cancers have attracted extensive attention and have been shown to be involved in oxidative stress response and carcinogenesis. Nevertheless, the roles of lncRNA AL033381.2 in regulating the development and progression of HCC still remain unclear. The purpose of our study was to evaluate the potential effects and molecular mechanisms of AL033381.2 that may be involved in oxidative stress response in HCC. Using bioinformatics analyses based on the TCGA database, we screened and identified a novel lncRNA AL033381.2 in HCC, which may be involved in oxidative stress responses. qRT-PCR analysis revealed that AL033381.2 is upregulated in HCC tissues. Through *in vitro* and *in vivo* experiments, we found that AL033381.2 dramatically facilitates the growth and metastasis of HCC. Mechanistically, RNA pull-down experiments, mass spectrometry, PathArray™, and RIP were used to determine that AL033381.2 binds to PRKRA and may be involved in AL033381.2-mediated oncogenic functions in HCC cells. Moreover, rescue experiments demonstrated that PRKRA overexpression rescues the abilities of HCC cell proliferation, migration, and invasion that were affected by AL033381.2 knockdown. Furthermore, we produced a nanoparticle-based siRNA delivery system and tested its therapeutic effects *in vivo*. The results showed that the *in vivo* growth rate of the tumors treated with the nanoparticle/AL033381.2 siRNA complexes was dramatically lower than those treated with the nanoparticle/scramble siRNA complexes. Taken together, our results suggest that the novel lncRNA AL033381.2 may be involved in oxidative stress response by targeting oxidative stress-related genes in HCC. AL033381.2 plays vital oncogenic roles in HCC progression and may be a novel therapeutic marker for HCC diagnosis and treatment.

## 1. Introduction

Hepatocellular carcinoma (HCC) is one of the major causes of cancer mortality around the world, and the occurrence of HCC continues to increase in China [1, 2]. As most HCC patients are commonly diagnosed at the advanced stage, and effective therapies and molecular targeted drugs are lacking, the prognosis of HCC patients remains poor [3, 4]. In recent years, a growing body of research has focused on targeted therapy for HCC [5]. The pathogenesis of HCC is a multistep process that is related to the gradual accumulation of genetic changes that accurately locate various cellular and molecular events, such as oxidative stress, endoplasmic reticulum stress, and abnormal cell cycles [6]. Oxidative stress is considered to play a crucial role in the initiation and promotion of carcinogenesis, and it can accelerate the progression of HCC through endogenous or exogenous injury and excessive production of reactive oxygen species (ROS) and active nitrogen (RNS), as well as reduced antioxidant defense [7]. More specifically, oxidative stress injury can affect the expression of cell survival genes, and its products promote the growth and differentiation of normal cells and eventually lead to the reduction of cell apoptosis and the formation of tumor cells [8]. Therefore, the level of oxidative stress can be a promising predictor of HCC diagnosis and treatment. Hence, it is crucial to clarify the mechanism of HCC progression and identify the valuable therapeutic targets for HCC.

Increasing evidence has demonstrated that several lncRNAs that are nonprotein-coding RNAs with a length of more than 200 nucleotides can be induced by oxidative stress, and thus, they are considered to be potential therapeutic targets in various cancers [9, 10]. In recent years, extensive evidence has revealed that lncRNA expression profiles are dysregulated in multiple malignancies and play a vital role in facilitating cancer progression through various molecular mechanisms [11]. LncRNAs are associated with regulating gene expression, chromatin remodeling, transcription control, splicing regulation, mRNA stabilization, microRNA processing, and protein stability maintenance [12]. Therefore, lncRNAs play vital roles in tumor growth, invasion, and metastasis [13]. Nevertheless, numerous lncRNAs have yet to be functionally characterized. Hence, a comprehensive understanding of the roles of lncRNAs in the occurrence and development of HCC will help to enrich our knowledge of the molecular mechanisms of HCC progression and also provide new insights into the development of therapeutic for HCC.

We identified oxidative stress-responsive lncRNA AL033381.2, which is a newly discovered lncRNA involved in tumor progression. In our study, we first report that AL033381.2 is notably elevated in HCC tissues, thereby implying that AL033381.2 plays a tumor-promoting role in HCC progression. Additionally, AL033381.2 enhances the abilities of HCC cell proliferation, migration, and invasion by regulating PRKRA. Moreover, we investigated the potential of AL033381.2 siRNA as a possible therapeutic target in HCC using a PLGA-based nanoparticle delivery system and tested its therapeutic effect *in vivo*. Our findings suggest that AL033381.2 can be potentially utilized as a diagnostic molecular biomarker and novel therapeutic target for HCC patients.

## 2. Materials and Methods

### 2.1. RNA-Sequencing Data Download and Analysis

For liver hepatocellular carcinoma (LIHC), the TCGA database [14] contains 374 samples with available data, including 50 samples with paired tissue (cancer and normal) RNA-sequencing (RNA-seq) data. A total of 317 patients were sampled with RNA-seq data and pathological data. Statistically significant differentially expressed lncRNAs (DElncRNAs) were screened out by R language analysis. The cut-off value was ∣log_2_FC (fold change) | >1 and FDR (false discovery rate) < 0.05.

### 2.2. Cell Culture and Clinical Specimens

Hep3B, Huh-7, HepG2, and SK-HEP-1 cell lines were obtained by the Cell Bank of the Chinese Academy of Sciences, which were authenticated by STR profiling. Cells were maintained in DMEM supplement with 10% FBS (Gibco) and cultured at 37°C under 5% CO_2_.

Besides, matched pairs of fresh HCC tissues and adjacent normal tissue samples (*n* = 30) from HCC patients were collected from January 2020 to January 2021 for Western blot analysis, with informed consent. Our study was approved by the Institutional Research Ethics Committee of the Affiliated Hospital of Nantong University.

### 2.3. Cell Transfection

The recombinant lentivirus of lncRNA AL033381.2 knockdown (shAL033381.2), negative control (shCtrl), and lentiviruses expressing PRKRA (LV-PRKRA) were synthesized by GeneChem (Shanghai). Hep3B and Huh-7 cells were infected with lentivirus at a MOI of 10 using Eni.S+polybrene. The target sequences of shAL033381.2 are as follows: 5′-GGAAAGAATAGTAGACATAATAGC-3′ (forward) and 5′-GAGCCGACACGGGTTAGGATCC-3′ (reverse).

### 2.4. Fluorescence In Situ Hybridization (FISH)

The subcellular localization of AL033381.2 in cells was tested by the FISH kit (RiboBio) following manufacturer's instruction, which was employed as previously described [15]. The AL033381.2 probe for FISH is 5′-CACGACTCTGGCAAGGTGAT-3′. The fluorescence was detected and photographed under a laser confocal microscope.

### 2.5. Immunohistochemistry (IHC)

The IHC staining assay was implemented as previously described [16]. Caspase-3 was detected with primary antibody (Abcam, ab184787) at 1 : 2400 dilution; E-cadherin was detected with primary antibody (Proteintech, 20874-1-AP) at 1 : 1800 dilution; Ki67 was detected with primary antibody (Abcam, ab15580) at 1 : 9600 dilution; MMP2 was detected with primary antibody (Proteintech, 10373-2-AP) at 1 : 100 dilution; MMP-9 was detected with primary antibody (CST, #13667) at 1 : 50 dilution; N-Cadherin was detected with primary antibody (Abcam, ab18203) at 1 : 600 dilution; PCNA was detected with primary antibody (CST, #2586) at 1 : 200 dilution; and PRKRA was detected with primary antibody (Affinity Biosciences, DF7334) at 1 : 500 dilution.

### 2.6. Quantitative Real-Time PCR

Total RNA was extracted by TRIzol (Invitrogen), which was then subjected to reverse transcriptase reaction with M-MLV reverse transcriptase (Takara). qPCR was carried out by SYBR Master Mixture (TaKaRa) and conducted using the LightCycler 480 II Detection System (Roche). The relative RNA levels were calculated by the 2^−ΔΔCt^ method, and GAPDH was applied for internal control. Primer sequences are listed: AL033381.2, 5′-CTGTAAGAAGTAAGGTCGGG-3′ (forward) and 5′-GCGTCCTCCTCCATAAGAT-3′ (reverse).

### 2.7. Western Blot Analysis

Western blot was conducted according to the previous protocol [17]. The primary antibodies were diluted to 1 : 500 for MMP9 (CST, #13667); diluted to 1 : 1000 for PRKRA (Affinity Biosciences, DF7334), P-eIF2*α* (CST, #3398), PKR (Abcam, ab32052), UBE2I (Abcam, ab75854), P-p53 (Abcam, ab33889), and MMP2 (CST, #40994); diluted to 1 : 2000 for N-cadherin (Proteintech, 22018-1-AP); and diluted to 1 : 5000 for eIF2*α* (CST, #5324), E-Cadherin (Proteintech, 20874-1-AP), and *β*-actin (Santa Cruz, sc-69879). Then, secondary antibodies were diluted to 1 : 10000 for Rabbit IgG (CST, #7074) and Mouse IgG (CST, #7076). The protein bands were visualized using the ECL detection kit (ECL, Thermo).

### 2.8. Cell Proliferation Assay

For cell counting assay, lentivirus-infected (shCtrl and shAL033381.2) cells were seeded at 96-well plates and cultured with 3000 cells/well. The plate was then tested by Celigo Image Cytometer (Nexcelom) for five days, and the proliferation curve was then created. For MTT assay, lentivirus-infected (shCtrl and shAL033381.2) cells were seeded into 96-well plates at 2 × 10^3^ cells/well and incubated for 5 days at 37°C. Subsequently, 20 *μ*L MTT solution (5 mg/mL) was added to each well and cultured at 37°C for 4 h. Cell viability was detected at the absorbance of 490 nm. For EdU assay, the positive cells in each group were counted and analyzed under the fluorescence microscope after using Cell-LightTM EdU Apollo567 kit (Ribo) in vitro according to manufacturer's instruction.

### 2.9. Colony Formation Assay

Cells were plated in 6-well plates with 5% CO_2_ at a density of 1000 cells/dish at 37°C. Two weeks later, colonies were fixed with 4% paraformaldehyde for 30 minutes and stained for 10 minutes with crystal violet. All colonies were washed several times with ddH_2_O, dried, and photographed.

### 2.10. Transwell Assay

Cell migration or invasion abilities were conducted by Transwell chambers (Corning, 8 *μ*m pore size) uncoated or coated with Matrigel, respectively. Firstly, 1 × 10^5^ cells per well suspended in 100 *μ*L FBS-free culture medium was seeded to the upper chamber, with a lower chamber filled with 600 *μ*L 30% FBS culture medium. After 24 hours, the filters were fixed and stained. In each chamber, the field of view was randomly selected for microscope photography, and cell number was calculated.

### 2.11. Flow Cytometry

Cells were seeded in six-well plates for cell apoptosis and cell cycle analyses and cultured overnight until reaching 70%-80% confluency. For cell apoptosis, cells were collected and stained with 10 *μ*L Annexin V-APC (eBioscience) and incubated in darkness for 15 minutes. For cell cycle, cells were resuspended and stained with PI (Sigma, 50 ng/mL) and RNase (Thermo Fisher Scientific, 10 ng/mL) for 20 minutes in darkness. Finally, cells were analyzed with Flow Cytometer (BD, C6 PLUS). Data analysis was performed by using the Novo Express software.

### 2.12. Tumor Xenograft Experiment

Huh-7 cells (1 × 10^7^) were injected subcutaneously into the right flank of BALB/c nude mice (4-week-old). Tumor sizes and mice weights were detected every three days. Tumor volume (mm^3^) was determined: tumor volume = width^2^ × length/2. Forty-five days after cell injection, the mice were euthanized, and the tumor tissues were weighed. Ethical approval for the animal experiments was obtained from the Animal Ethics Committee of Affiliated Hospital of Nantong University.

### 2.13. RNA Immunoprecipitation Assay (RIP)

RIP experiments were employed using the Magna RIP RNA-Binding Protein Immunoprecipitation Kit following manufacturer's protocol. Antibodies against snRNP70 and normal IgG were, respectively, used as positive and negative controls. qRT-PCR was utilized to determine the RNA enrichment of AL033381.2, which was normalized to the amount of the enriched U1 RNA. Then, the qRT-PCR products were collected for agarose gel electrophoresis, and the existence of AL033381.2 and PRKRA was directly observed.

### 2.14. RNA Pull-down Assay and Mass Spectrometry Analysis

AL033381.2 was transcribed using T7 RNA polymerase in vitro, followed by purification with an RNeasy Plus mini kit. Purified RNAs were labeled with Biotin RNA labeling Mix. Proteins extracted from cells were mixed with biotinylated AL033381.2 or antisense RNA probe that was synthesized by GeneChem and incubated with streptavidin agarose beads. The related proteins were separated by gel electrophoresis and then visualized by silver staining. LncRNA-binding proteins were eluted and subjected to mass spectrometry. LC-MS/MS data were analyzed for protein identification and quantification using PEAKS Studio 8.5. Finally, the eluted proteins were analyzed by Western blotting.

### 2.15. Preparation and Characterization of Nanoparticle/siRNA Complexes

As previously described [18], PLGA nanoparticles were produced by oil-in-water solvent evaporation technology with minor modifications. First, a 10% polymer solution was formed by dissolving 100 mg PLGA in 1 mL dichloromethane. Three milliliters of 7% polyvinyl alcohol aqueous solution was then added to the polymer solution and emulsified by sonication for 120 s. Subsequently, the emulsion was added into 50 mL of a 1% polyvinyl alcohol aqueous solution. These mixtures were sonicated for 180 s and stirred for 24 h to vaporize the dichloromethane. After that, the nanoparticle suspension was washed, centrifuged at 13,000 rpm for 5 min, and resuspended in ddH_2_O. Approximately 100 *μ*L of the nanoparticle aqueous solution was mixed with 2 *μ*L of polyethyleneimine polymer aqueous solution to form polyethyleneimine-modified nanoparticles. Then, we performed a gel retardation assay to test the best proportion of nanoparticles and siRNA. Subsequently, the polyethyleneimine-modified nanoparticle suspension was added to the siRNA solution of polymer nitrogen and RNA phosphate, gently mixed, and cultured for 15 min to yield nanoparticle/siRNA complexes. Finally, the ultrastructure of the nanoparticle/siRNA complexes was examined by scanning electron microscopy. The average hydrodynamic diameter of nanoparticle/siRNA complexes was measured by dynamic light scattering. Finally, Zetaplus was used to detect the zeta potential of the complexes at 25°C with a 90° scattering angle.

### 2.16. In Vivo Tumor Inhibition of AL033381.2 siRNA-Loaded Nanoparticles

Huh7 cells were inoculated into the armpit of 18–22 g nude mice to establish a tumor xenograft model. The animals were weighed and randomly divided into two groups, namely, nanoparticle/scramble siRNA complexes and nanoparticle/AL033381.2 siRNA complexes, when the tumor volume of the animals reached about 50 mm^3^. Subsequently, the tumor sizes were observed with a Vernier caliper every other day and calculated as Volume = Width^2^ × Length/2. The mice were euthanized 16 days later, and tumors were dissected and weighed. The animal ethical statement was previously described.

### 2.17. Statistical Analysis

All statistical analysis was conducted using SPSS 25.0. All data are presented as means ± standard deviation from at least 3 independent experiments. Then, Student's *t*-test (two-tailed), chi-squared tests, and one-way ANOVA were performed to compare the significance of differences between groups. Statistically significance was chosen as *P* < 0.05.

## 3. Results

### 3.1. LncRNA AL033381.2 Is Upregulated in HCC Tissues

To investigate novel lncRNAs that play a key role in HCC, we analyzed the DElncRNAs between tumor and normal tissues in the TCGA database and identified AL033381.2 as one of the highly upregulated candidates in HCC that has not been reported and studied to date (Figures 1(a) and 1(b)). Then, bioinformatics analysis of TCGA data revealed that AL033381.2 expression is highly upregulated in liver cancer tissues relative to paired adjacent normal tissues (Figures 1(c)–1(e), *P* < 0.05). To further assess the roles of AL033381.2 in HCC, we evaluated the expression level of AL033381.2 in a cohort of 30 HCC tissue samples and matched adjacent normal samples by qRT-PCR analysis. Our results showed that the AL033381.2 expression level is upregulated in HCC tissues compared to paired adjacent normal tissues (Figure 1(f), *P* < 0.001). Moreover, as shown in Supplementary Figure S1, qRT-PCR analysis showed that AL033381.2 is expressed in Hep3B, Huh-7, HepG2, and SK-HEP-1 cell lines.

To investigate the mechanism by which AL033381.2 acts as an oncogenic lncRNA by driving tumorigenesis in HCC, we analyzed the subcellular distribution by FISH. The results indicated that AL033381.2 exhibited a predominantly cytoplasmic localization in Hep3B and Huh-7 cells (Figure 1(g)), which suggests that AL033381.2 might exert regulatory functions in the cytoplasm.

We also performed the Mann-Whitney *U* test to analyze the significance of different expression levels of AL033381.2 in various clinical data at different levels. As we can see from the significance index of the test, the expression of AL033381.2 was markedly different in the cancer tissues of patients with different T stages and pathological stages at the significance level of 0.05. It is suggested that the AL033381.2 expression level may be correlated to T stage and pathological stage (Table 1). Moreover, Spearman's test was used to statistically analyze the correlation between the AL033381.2 expression level in cancer tissues and clinical data to preliminarily explore the potential role of these clinical data in the genesis and development of liver cancer. The significance index of the test indicated that the AL033381.2 expression level in tumor tissues was remarkably correlated to the pathological stage of the patients at a significance level of 0.05, suggesting that the expression level of this gene might be used as an indicator for clinical diagnosis of the pathological stage. The AL033381.2 expression was positively associated with the pathological stage level, suggesting that the AL033381.2 expression level gradually increased with the progression of liver cancer (Table 2).

### 3.2. Knockdown of AL033381.2 Suppresses Cell Proliferation, Migration, and Invasion and Promotes Apoptosis

The roles of AL033381.2 in cell proliferation, cell viability, colony formation ability, cell migration, and invasion abilities were analyzed by MTT, Celigo Imaging Cytometry System, colony formation, EdU, and Transwell assays, respectively. First, compared to the shCtrl group, mRNA expression of AL033381.2 in Hep3B and Huh-7 cells was downregulated after transduction with lentivirus shAL033381.2 (Figures 2(a) and 2(c)). MTT assays revealed that the viability of Hep3B and Huh-7 cells was notably reduced in the shAL033381.2 group compared with the shCtrl group (Figures 2(b) and 2(d)). Furthermore, Celigo cell counting assays revealed that cell proliferation was remarkably suppressed in the shAL033381.2 group compared with the shCtrl group in Hep3B and Huh-7 cells (Figures 2(e) and 2(f)).

Additionally, colony formation assays showed that fewer colonies were formed by Hep3B and Huh-7 cells in the shAL033381.2 group compared with the shCtrl group (Figure 3(a)). Moreover, we assessed the effects of AL033381.2 on the abilities of HCC cell migration and invasion by Transwell assays. Our results demonstrated that the number of migrating and invasive cells was markedly reduced upon transfection with lentivirus shAL033381.2 compared to the shCtrl group (Figures 3(b) and 3(c)). Additionally, EdU proliferation assays were performed to assess the effects of AL033381.2 on the DNA replication of HCC cells. We found that cell proliferation was inhibited after transfection with lentivirus shAL033381.2 in Hep3B and Huh-7 cells (Figures 3(d) and 3(e)).

To further explore the mechanisms of AL033381.2 on cell proliferation, we conducted flow cytometry to detect the distribution of the cell cycle and the apoptosis rate of HCC cells transfected with lentivirus shAL033381.2. Cell cycle analysis indicated that the cell percentage in the G0/G1 phase was obviously elevated, and the percentage of Hep3B and Huh-7 cells in the S phase markedly decreased after transfection with lentivirus shAL033381.2 (Figures 3(f) and 3(h)). Furthermore, we found that the rate of apoptosis in Hep3B and Huh-7 cells increased after transfection with lentivirus shAL033381.2 (Figures 3(g) and 3(i)). Collectively, these results suggest that AL033381.2 plays a pivotal role in regulating HCC pathogenesis.

### 3.3. Knockdown of AL033381.2 Suppresses Tumor Growth In Vivo

To further verify the roles of AL033381.2 in tumor growth of HCC cells in vivo, we calculated the weight and volume of tumors using the xenograft model. Our results revealed that the shAL033381.2 group showed dramatically reduced tumor volume and weight compared with those in the shCtrl group (Figures 4(a)–4(c)). IHC staining revealed reduced expression of Ki-67, PCNA, caspase-3, E-cadherin, N-cadherin, MMP2, and MMP9 in the shAL033381.2 group, while H&E staining indicated more extensive focal necrosis in the shAL033381.2 group (Figure 4(d)). In parallel, the elevated expression level of E-cadherin and reduced expression level of N-cadherin, MMP2, and MMP9 at the protein levels in the Hep3B and Huh-7 cells were found to be associated with the shAL033381.2 group (Figure 4(e)). Our above results confirm that AL033381.2 plays a vital role in *in vivo* HCC tumorigenesis.

### 3.4. AL033381.2 Binds to the PRKRA Protein

Bioinformatics analysis was performed to predict the secondary structure of AL033381.2 (Supplementary Figure S2). To further elucidate that the molecular mechanism of AL033381.2 involves tumor promotion, we performed an RNA pull-down assay using biotin-labeled RNA to identify potential proteins binding to AL033381.2 in Huh-7 cells. The remaining bands specific to AL033381.2 were subjected to LS/MS mass spectrometry (Figures 5(a) and 5(b)). According to the list of differential genes in the results of mass spectrometry (Supplementary Figure S3, S4), the subcellular localization of genes was matched through the IPA database, and the genes identified as cytoplasmic were selected to draw a network diagram together with cell proliferation and apoptosis (Figure 5(c)). The direct interaction between AL033381.2 and its RNA-binding proteins was further confirmed by Western blotting of Huh-7 cell lysate using antibodies against STAU1, PRKRA, PRDX2, RNH1, KRT8, and ETFB (Supplementary Figure S5). Then, RIP assay followed by qRT-PCR demonstrated that the enrichment of AL033381.2 precipitated by antibodies against PRKRA, PRDX2, RNH1, and ETFB dramatically increased compared with the control IgG in Huh-7 cells (Figure 5(d)). Consistently, Western blotting followed by RIP assays confirmed the capability of PRKRA, PRDX2, RNH1, and ETFB to bind to AL033381.2 in Huh-7 cells (Figure 5(e)). Moreover, we employed an additional RNA pull-down assay followed by Western blotting using the PRKRA antibody to determine the interaction of AL033381.2 with PRKRA. The results showed that labeled AL033381.2, but not antisense, indicated the ability to specifically retrieve PRKRA from cell extracts (Figure 5(f)). Furthermore, the RIP assay verified that AL033381.2 was precipitated by the PRKRA antibody (Figure 5(g)). In addition, to explore the effects of AL033381.2 on PRKRA, we assessed the protein expression level of PRKRA in Huh-7 cells transfected with shAL033381.2 or shCtrl lentivirus. Western blotting confirmed that PRKRA protein expression notably decreased with shAL033381.2 transfection (Figure 5(h)). The above findings suggest that AL033381.2 interacts with PRKRA protein, which in turn contributes to the regulation of HCC progression.

### 3.5. Restoration of PRKRA Rescues AL033381.2 Knockdown-Mediated Suppression of Cell Proliferation, Migration, and Invasion

Following the determination that the downstream targets of AL033381.2 are PRKRA, PRDX2, RNH1, and ETFB, we performed *in vitro* experiments to explore whether these genes could mediate the inhibitory effects of AL033381.2 knockdown. According to Celigo cell counting assays, only PRKRA overexpression could partially abrogate the inhibition of the cell proliferation induced by AL033381.2 knockdown compared with the controls (Figure 6). To further investigate whether AL033381.2 functions in a PRKRA-mediated manner in HCC progression, we conducted additional experiments to verify the recovery effects of PRKRA overexpression lentivirus and lentivirus shAL033381.2 coinfected HCC cells. MTT and colony formation assays demonstrated that PRKRA overexpression partially abrogated the decreased viability and clonogenicity of Hep3B and Huh7 cells caused by AL033381.2 knockdown (Figures 7(a)–7(d)). Furthermore, Transwell assays showed that knockdown of AL033381.2 suppressed the migration and invasion of Hep3B and Huh7 cells, whereas PRKRA overexpression partially abolished these effects (Figures 7(e) and 7(f)). Meanwhile, EdU assays indicated that overexpressing PRKRA rescued the reduction in the proliferation of Hep3B and Huh7 cells caused by AL033381.2 knockdown (Figures 7(g) and 7(h)).

To further confirm whether AL033381.2 is related to the EMT pathway via modulating PRKRA, we transfected HCC cells with lentivirus shAL033381.2 and PRKRA overexpression lentivirus. As presented in Figure 7(i), shAL033381.2 upregulated E-cadherin expression and downregulated N-cadherin, MMP2, and MMP9 expression in Hep3B and Huh-7 cells, whereas overexpression of PRKRA abolished these effects. Our results consistently indicated that AL033381.2 inhibits HCC progression via activation of PRKRA.

### 3.6. In Vivo Antitumor Efficacy of Nanoparticle/siRNA Complexes

The morphology of the nanoparticle/siRNA complexes was analyzed by SEM, which presented representative images of the empty nanoparticles and nanoparticle/siRNA complexes (Figure 8(a)). As shown in Figure 8(b), the hydrodynamic diameter of complexes demonstrated that the mean diameter of the empty nanoparticles and nanoparticle/siRNA complexes was ~103 nm and 108 nm, respectively. A gel retardation assay showed that nanoparticles containing siRNA exhibited the best retarding effect when the *N*/*P* ratio was 6 : 1 (Figure 8(c)). Then, we performed a slower sustained release profile of siRNA from the nanoparticle/siRNA complexes, and we observed that about 90% of the loaded siRNA were released within 27 days (Supplementary Figure S6). The zeta potential of the empty nanoparticles and nanoparticle/siRNA complexes was about −15.2 mV and 23.1 mV, respectively. Moreover, we performed flow cytometry to test the transfection efficiency of nanoparticle/FAM-siRNA complexes. FAM-siRNA was delivered into the Huh7 cells, with a transfection efficiency of about ~70% (Figures 8(d) and 8(e)), indicating that the nanoparticle/siRNA complexes possess good transfection efficiency in Huh7 cells.

Furthermore, to evaluate the *in vivo* antitumor efficacy of the nanoparticle/AL033381.2 siRNA complexes, we calculated the weight and volume of tumors after different formulations were administrated into nude mice. The mice treated with nanoparticle/AL033381.2 siRNA complex group exhibited lower tumor volume and weight compared with the scrambled group, thus demonstrating that AL033381.2 siRNA-loaded nanoparticles presented better anticancer efficacy (Figures 8(f)–8(h)). In addition, we assessed the expression of AL033381.2 at the mRNA level from tumor samples of mice treated with several complexes using qRT-PCR, which indicated that AL033381.2 expression in mice treated with the nanoparticle/AL033381.2 siRNA complex group was dramatically lower than those in the scrambled group (Figure 8(i)). The above results demonstrated that AL033381.2 may potentially be utilized as a therapeutic target, and the nanoparticle drug delivery system can be an effective therapeutic alternative.

## 4. Discussion

Emerging research has revealed that the vital roles of lncRNAs in tumorigenesis and tumor progression in several cancers have attracted increasing attention [19]. The accumulation of lncRNAs has been associated with tumorigenesis, including HCC [20, 21]. For instance, Wen et al. showed that the lncRNA ANCR accelerates the EMT and migration and invasion of HCC cells by modulating HNRNPA1 [22]. Zhang et al. demonstrated that lncRNA UPK1A-AS1 indicates poor prognosis in HCC and interacts with EZH2 to promote cell growth [23]. Most recently, Zhang et al. have shown that LIN28B-AS1 is associated with IGF2BP1 and promotes human HCC cell progression *in vitro and in vivo.* [24]. Although accumulating studies have shown the potential oncogenic roles of lncRNAs in a variety of cancers [25, 26], AL033381.2 is still a novel lncRNA molecule, and its role in tumor progression remains unclear.

In this study, we attempted to determine the expression profile and biological effects of AL033381.2 in HCC and elucidate its potential molecular mechanism. Then, we identified the differentially expressed lncRNAs in the TCGA database in both cancer tissues and normal tissues by integrating bioinformatics analysis. Our results indicated that in liver cancer, AL033381.2 is markedly upregulated and closely correlated to some clinicopathological parameters, including T stage, TNM stage, and pathological grade. To further verify the sequencing results, we investigated the expression of AL033381.2 using qPCR in a cohort of 30 HCC tissues and corresponding normal tissues, and we found that AL033381.2 expression was observably increased in HCC tissues compared to matched normal tissues. In addition, numerous studies have revealed that owing to the involvement of lncRNAs in the regulation of tumor-related genes, lncRNAs are involved in several cell processes, including cell proliferation, growth, differentiation, and apoptosis [27]. Based on our experimental findings, AL033381.2 consistently acts as an oncogene that promotes the proliferation and metastasis of HCC cells *in vivo* and *in vitro*.

Epithelial-to-mesenchymal transition (EMT) is a biological process wherein epithelial cells lose the requirements for physical contact with adjacent cells and acquire mesenchymal characteristics, including enhanced migratory and invasive behaviors [28]. In particular, lncRNAs positively regulate the EMT process in HCC [29]. Here, we demonstrate that AL033381.2 promotes EMT progression in HCC cells and thus could be utilized as a new target for molecular targeted therapy of HCC. Consequently, the abnormal expression and crucial functions of AL033381.2 in HCC prompted us to further elucidate its potential regulatory mechanism.

LncRNAs exert their functions in multiple mechanisms, including scaffolding nuclear and cytoplasmic complexes, gene expression modulation, and cotranscriptional regulations [30]. Moreover, the function of lncRNAs is often related to their subcellular location [31]. Cytoplasmic lncRNAs may be involved in regulating protein stability and translational modification [32]. In this study, to further evaluate the molecular mechanisms of AL033381.2 in promoting HCC tumorigenesis, we first performed FISH assays, which indicated that AL033381.2 is predominantly cytoplasmic and possibly exerts in biological function at the posttranscriptional level. Mechanically, RNA pull-down and mass spectrometry analysis finally identified PRKRA as one of several proteins bound to AL033381.2. Moreover, we demonstrated that PRKRA interacts with AL033381.2 using RIP and RNA pull-down assays. PRKRA, which is a known cellular protein activator of PKR kinase [33], participates in microRNA processing and interacts with members of the RNAi pathway such as Dicer and Ago2 [34]. A previous study has shown that PRKRA is upregulated in lung adenocarcinoma [35]. Recent studies have also demonstrated that treatment with siPRKRA plus oxaliplatin imparts a significant antitumor effect on mucinous ovarian cancer cells [33]. Furthermore, in our study, functional analyses indicated that AL033381.2 knockdown markedly suppresses HCC cell proliferation and metastasis and that this effect is partially rescued by simultaneous PRKRA overexpression. Additionally, our studies have shown that AL033381.2 could promote the EMT pathway by regulating PRKRA.

Recent studies have shown that nonviral vectors, nanoparticle gene vectors in particular, have low toxicity and biodegradability [36]. In our study, PLGA nanoparticles were prepared as siRNA transfection vectors. The growth rate of AL033381.2 siRNA-loaded nanoparticle-Huh-7 tumors in nude mice was notably slower than the control group, indicating that nanoparticle/AL033381.2 siRNA complexes significantly inhibit tumorigenesis *in vivo* and thus impart positive therapeutic effects.

## 5. Conclusions

This is the first report that shows that lncRNA AL033381.2 imparts carcinogenic effects on HCC by interacting with PRKRA. Nanoparticle/AL033381.2 siRNA complexes also exhibit favorable therapeutic effects in vivo and have the potential to become a novel therapeutic target worthy of further investigation. This study provides a novel investigation of the potential therapeutic target of AL033381.2 and provides a better understanding of the pathogenesis and molecular treatment strategies of HCC. Consequently, further research is needed to elucidate the regulatory mechanisms of the AL033381.2/PRKRA axis and identify particular targets for therapeutic applications to HCC.

## Figures and Tables

**Figure 1:** LncRNA-AL033381.2 expression is upregulated in HCC tissues. (a, b) Heatmaps and volcano plots of the differential expressed lncRNAs between LIHC tissues (*n* = 374) and normal controls (*n* = 50) in TCGA, including the increased levels of AL033381.2. (c) The differential expression of AL033381.2 in the original data of each TCGA RNA-seq sample can be represented by a line graph. The vertical axis is the original data of the expression level of each sample, and the horizontal axis is the cancer tissue and normal tissue of the sample, with one broken line for each sample. (d) The differential expression of AL033381.2 in cancer (*n* = 50) and normal tissue samples (*n* = 50) can be demonstrated by log_2_FC, *P* value, and FDR in the TCGA database. (e) Differential gene expression can also be shown in a histogram. The vertical axis is the log_2_FC, and the horizontal axis is different samples, and the log_2_FC of each sample is represented by a column diagram. (f) The relative expression of AL033381.2 between HCC samples and corresponding normal tissues was compared by qRT-PCR analysis (*n* = 30). (g) The subcellular location of AL033381.2 in Hep3B and Huh7 cells was determined by FISH analysis after transfection. Nuclei were stained with DAPI. U6 or GAPDH was used as nuclear and cytosolic markers, respectively.

**Figure 2:** Knockdown of AL033381.2 suppressed the proliferation of HCC cells. (a, c) The mRNA expression level of AL033381.2 in Hep3B and Huh-7 cells was determined by qRT-PCR analysis. (b, d) The proliferative rates of Hep3B and Huh-7 cells were assessed by MTT assay. (e, f) After infection of lentivirus shAL033381.2 or shCtrl, celigo cell counting assay was employed to assess the viability of Hep3B and Huh-7 cells. ^∗^*P* < 0.05; ^∗∗^*P* < 0.01; ^∗∗∗^*P* < 0.001.

**Figure 3:** Knockdown of AL033381.2 suppressed the proliferation, migration, and invasion of HCC cells and induced cell apoptosis and regulates the cell cycle process. (a) Colony formation assay was employed to examine the effects of AL033381.2 knockdown on the proliferation of Hep3B and Huh-7 cells. (b, c) Transwell assay was employed to measure the effects of AL033381.2 knockdown on cell migration and invasion of Hep3B and Huh-7 cells. (d, e) EdU incorporation assay was used to evaluate the abilities of DNA replication on Hep3B and Huh-7 cells after infection of lentivirus shAL033381.2 or shCtrl. (f–i) The apoptosis and cell cycle distribution of Hep3B and Huh-7 cells were analyzed by flow cytometry after shAL033381.2 or shCtrl lentivirus transfection. ^∗^*P* < 0.05; ^∗∗^*P* < 0.01.

**Figure 4:** Knockdown of AL033381.2 inhibited tumor growth in vivo. (a) Typical images of xenograft tumors formed by Huh-7 cells transfected with shCtrl or shAL033381.2 from each group of mice. (b, c) Tumor volume and tumor weight in each group of mice. (d) Typical H&E staining and IHC staining images of Ki-67, PCNA, Caspase 3, E-cadherin, N-cadherin, MMP2, and MMP9 in xenograft tumor tissues from each group of mice. ^∗∗^*P* < 0.01. (e) The expression of E-cadherin, N-cadherin, MMP2, and MMP9 at the protein level in transfected cells with shCtrl or shAL033381.2 were examined by Western blot analysis.

**Figure 5:** AL033381.2 interacts with PRKRA. (a, b) The specific biotin-labeled AL033381.2 probe was added to the cell lysate, and the precipitated proteins were resolved by SDS-PAGE and then stained with silver. The AL033381.2 probe was analyzed by using SDS-PAGE. The antisense of AL033381.2 and the beads serve as the control. The AL033381.2-specific bands (red rectangle) were excised and analyzed using mass spectrometry. (c) IPA analysis identified the genes located in the cytoplasm were associated with cell proliferation and apoptosis. (d) RIP assay showed that STAU1, PRDX2, ETFB, PRKRA, KRT8, and RNH1 interacted with AL033381.2 in Huh-7 cells by RT-qPCR analysis. (e) Western blot results exhibited the capability of PRKRA, PRDX2, RNH1, and ETFB binding to AL033381.2 in Huh-7 cells. (f) RNA pull-down assay was conducted in Huh-7 cells using biotinylated AL033381.2 or antisense RNA probe transcribed in vitro and measured by western blots. (g) RIP assay was employed in Huh-7 cells using an antibody against PRKRA to determine AL033381.2 RNA enrichment in immunoprecipitated complexes with IgG as a negative control. (h) Western blot analysis was applied to determine the protein level of PRKRA after transfection of the cells with shAL033381.2 or shCtrl.

**Figure 6:** Overexpression of PRKRA rescued the cell proliferation caused by AL033381.2 knockdown in HCC cells. Celigo cell counting assay indicated that the proliferation of HCC cells was suppressed significantly in KD+NC group cells compared with NC+NC group cells, and overexpression of PRKRA (KD+OE1) rescued the inhibition of the cell proliferation induced by AL033381.2 knockdown. NC+NC group: normal target cells (Huh-7) and negative control lentivirus-infected cells (shCtrl); KD+NC group: shAL033381.2 lentivirus-infected cells (shAL033381.2) and overexpression of empty vector lentivirus-infected cells; KD+OE1 group: shAL033381.2 lentivirus-infected cells and the downstream gene PRKRA overexpressed lentivirus-infected cells; KD+OE2 group: shAL033381.2 lentivirus-infected cells and the downstream gene PRDX2 overexpressed lentivirus-infected cells; KD+OE3 group: shAL033381.2 lentivirus-infected cells and the downstream gene RNH1 overexpressed lentivirus-infected cells; KD+OE4 group: shAL033381.2 lentivirus-infected cells and the downstream gene ETFB overexpressed lentivirus-infected cells. ^∗∗∗^*P* < 0.001.

**Figure 7:** Overexpression of PRKRA rescued the inhibitory effects mediated by AL033381.2 knockdown in HCC cells. (a–h) The inhibitory functions of AL033381.2 silencing on cell viability, proliferation, migration, and invasion were measured by MTT (a, c), colony formation assays (b, d), Transwell (e, f), and EdU staining assays (g, h) in Hep3B and Huh-7 cells transfected with the PRKRA overexpressed lentivirus or control vector, respectively. (i) The expressions levels of E-cadherin, N-cadherin, MMP2, and MMP9 were detected by Western blot analysis in Hep3B and Huh-7 cells that were transfected with shCtrl, shAL033381.2, or shAL033381.2+PRKRA groups, respectively. ^∗^*P* < 0.05.

**Figure 8:** Characterization, transfection efficiency, and in vivo antitumor efficacy of nanoparticle/siRNA complexes. (a) Representative scanning electron microscopy images of the empty nanoparticles and nanoparticle/siRNA complexes; magnification 10,400x. (b) Hydrodynamic diameter distribution of the empty nanoparticles and nanoparticle/siRNA complexes. (c) A gel retardation assay of nanoparticle/siRNA complexes at different N/P ratios. (d, e) Representative fluorescent images, matched bright images, and transfection efficiency of Huh7 cells transfected with empty nanoparticles and nanoparticle/siRNA complexes. (f) The representative images of tumor growth in the subcutaneous xenograft model of Huh7 cells in nude mice. (g, h) In vivo antitumor results revealed the effects of tumor volume and weight after the treatment with nanoparticle/scramble siRNA complexes (scramble) and nanoparticle/AL033381.2 siRNA complexes (AL033381.2 siRNA). ^∗^*P* < 0.05. (i) The relative mRNA expression level of AL033381.2 between the scramble and AL033381.2 siRNA Huh7 cell lines.

**Table 1:** Analysis of the significant difference of AL033381.2 expression level in clinicopathologic characteristics.

Clinical parameters	AL033381.2 expression		Total	*P* value
	Low expression	High expression		
Pathological grade				
G1/2	149	83	232	0.119
G3/4	75	59	134	
Total	224	142	366	
T stage				
T1	121	60	181	0.032
T2	53	41	94	
T3/4	51	42	93	
Total	225	143	368	
TNM				
Stage I	115	56	171	0.011
Stage II	51	35	86	
Stage III/IV	46	44	90	
Total	212	135	347	

Statistical analyses were performed by the Mann-Whitney *U* test. ^∗^*P* value < 0.05 was considered statistically significant.

**Table 2:** Correlation analysis of clinicopathologic characteristics with AL033381.2 expression.

	AL033381.2 expression	T stage	Pathological grade
AL033381.2 expression			
Correlation coefficient	1.000	0.095	0.117
Significance (double tail)		0.070	0.029
T stage			
Correlation coefficient	0.095	1.000	0.981
Significance (double tail)	0.070		0.000
Pathological grade			
Correlation coefficient	0.117	0.981	1.000
Significance (double tail)	0.029	0.000	.

Statistical analyses were performed by Spearman's test. ^∗^*P* value < 0.05 was considered statistically significant.

## Data Availability

The data that support the findings of this study are available from the corresponding authors upon reasonable request.

## Supplementary Materials

Supplementary Materials Figure S1: the results of qRT-PCR showed that AL033381.2 was expressed in Hep3B, Huh-7, HepG2, and SK-HEP-1 cells. The relative mRNA expression (AL033381.2/GAPDH) was determined by the 2^−ΔΔCt^ method. Figure S2: the secondary structure of AL033381.2 (ENST00000603854) is shown as predicted by lnCAR (https://lncar.renlab.org). Figure S3: to exclude from antisense, mass spectrometry analysis showed the target gene list from AL033381.2 sense. Figure S4: mass spectrometry analysis of PRKRA binding to AL033381.2. Figure S5: Western blot analysis for RNH1, STAU1, ETFB, PRKRA, Peroxiredoxin2 (PRDX2), and Cytokeratin8 (KRT8) protein levels in Huh-7 cell lysates. Figure S6: in vitro cumulative release profiles of siRNA from the nanoparticle/siRNA complexes.
